The article "Thyroid Ultrasound Findings in Children from Three Japanese Prefectures: Aomori, Yamanashi and Nagasaki" was retracted in 2024. Reasons: duplicate publication; overlap with earlier publications; concerns about the data.

# Thyroid Ultrasound Findings in Children from Three Japanese Prefectures: Aomori, Yamanashi and Nagasaki

**DOI:** 10.1371/journal.pone.0083220

**Published:** 2013-12-23

**Authors:** Naomi Hayashida, Misa Imaizumi, Hiroki Shimura, Noriyuki Okubo, Yasushi Asari, Takeshi Nigawara, Sanae Midorikawa, Kazuhiko Kotani, Shigeyuki Nakaji, Akira Otsuru, Takashi Akamizu, Masafumi Kitaoka, Shinichi Suzuki, Nobuyuki Taniguchi, Shunichi Yamashita, Noboru Takamura, for the Investigation Committee for the Proportion of Thyroid Ultrasound Findings

**Affiliations:** 1 Department of Global Health, Medicine and Welfare, Atomic Bomb Disease Institute, Nagasaki University, Nagasaki, Japan; 2 Department of Radiation Medical Sciences, Atomic Bomb Disease Institute, Nagasaki University, Nagasaki, Japan; 3 Department of Clinical Studies, Radiation Effects Research Foundation, Nagasaki, Japan; 4 Department of Social Medicine, Hirosaki University Graduate School of Medicine, Hirosaki, Aomori, Japan; 5 Department of Emergency and Disaster Medicine, Hirosaki University Graduate School of Medicine, Hirosaki, Aomori, Japan; 6 Department of Endocrinology and Metabolism, Hirosaki University Graduate School of Medicine, Hirosaki, Aomori, Japan; 7 Department of Laboratory Medicine, Fukushima Medical University, Fukushima, Japan; 8 Department of Radiation Health Management, Fukushima Medical University, Fukushima, Japan; 9 Department of Thyroid and Endocrinology, Fukushima Medical University, Fukushima, Japan; 10 Radiation Medical Science Center for the Fukushima Health Management Survey, Fukushima Medical University, Fukushima, Japan; 11 Department of Clinical Laboratory Medicine, Jichi Medical University, Tochigi, Japan; 12 The First Department of Medicine, Wakayama Medical University, Wakayama, Japan; 13 Division of Endocrinology and Metabolism, Showa General Hospital, Tokyo, Japan; Kagoshima University Graduate School of Medical and Dental Sciences, Japan

## Abstract

Due to the likelihood of physical and mental health impacts following the unprecedented accident at the Fukushima Dai-ichi Nuclear Power Plant, the Fukushima prefectural government decided to conduct the Fukushima Health Management Survey to assist in the long-term health management of residents. This included thyroid ultrasound examination for all children in Fukushima. For appropriate evaluation of ultrasound screening of the thyroid, it is important to understand its reference data of thyroid findings in children in general. In order to analyze the frequencies of specific thyroid findings, we conducted ultrasound screening of the thyroid by the same procedures as used in Fukushima in 4,365 children, aged 3 to 18 years, from three Japanese prefectures. Overall, thyroid cysts were identified in 56.88% and thyroid nodules in 1.65% of the participants. Thyroid cysts and nodules with a maximum diameter of more than 5 mm were identified in 4.58% and 1.01%, respectively, and age-adjusted prevalences were 3.82% and 0.99%, respectively. Although the prevalence of cysts and nodules varied among the examination areas, no significant differences were observed among the three examination areas in the prevalence of cysts and nodules with a maximum diameter of more than 5 mm. Also, the prevalence of thyroid cysts and nodules, especially those with a maximum diameter of more than 5 mm, significantly increased with age, and showed a female predominance. We also identified ectopic thymus (1.95%), diffuse goiter (1.40%), ultimobranchial body (0.73%), lymph node swelling (0.21%) and thyroid agenesis (0.05%). This is the first ultrasound description of the age-adjusted prevalence of thyroid cysts and nodules, or of the prevalence of abnormalities other than cysts and nodules, such as ectopic thymus, in relation to age, in the general Japanese child population. We contend that this can provide relevant information for the Fukushima Health Management Survey and future population studies.

## Introduction

On March 11, 2011, a 9.0-magnitude earthquake (The Great East Japan Earthquake) struck the east coast of Japan, near Iwate, Miyagi and Fukushima Prefectures. The earthquake, together with the resulting tsunami, caused extensive damage to the Fukushima Dai-ichi Nuclear Power Plant (FNPP), such that a radioactive plume emanating from Units 1, 2, 3 and 4 of FNPP was dispersed into the atmosphere. The total quantity of radioactive materials released into the environment is estimated to be 10% [1.6×10^17^ Bq for ^131^I (half-life: 8.0 d) and 1.5×10^16^ Bq for ^137^Cs (30 y)] of that released following the accident at the Chernobyl Nuclear Power Plant (CNPP, 1.8×10^18^ Bq for ^131^I and 8.5×10^16^ Bq for ^137^Cs) [1], [2].

Due to the possible health impacts of this nuclear accident, the Fukushima prefectural government decided to conduct the Fukushima Health Management Survey to assist in the long-term health management of residents, and this is being carried out by Fukushima Medical University [3]. This survey consists of a basic survey to estimate the individual radiation exposure of residents, and four detailed surveys, including thyroid ultrasound examination, comprehensive health check-up, mental health and life-style survey, and a survey on pregnant women and nursing mothers [3]. The thyroid ultrasound examinations on March 11, 2011, targeting all prefectural inhabitants aged between 0 and 18 years (approximately 360,000 inhabitants), have received much attention, since it is well known that the incidence of childhood thyroid cancer increased after the Chernobyl accident [4], [5]. However, for a valid comparison of the results of the ultrasound screening of the thyroid, it is important to understand the normal ultrasound occurring in childhood, since ultrasound technology, including imaging quality, has dramatically advanced in recent years.

The prevalence of incidental thyroid abnormalities detected on ultrasound examinations in adults has been well documented [6]–[9]. However, few reports have studied the prevalence, spectrum of appearance, and management of ultrasound-detected findings in children [10], [11], except for the screening programs conducted around Chernobyl [4], [5]. Avula et al. conducted retrospective analysis of clinical and ultrasound findings in 287 Canadian children from 2006 to 2007, and detected incidental thyroid findings in 52 of them (18%) [10]. Among them, 35 were small (<4 mm) well-defined cysts, and nine were hypoechoic, solid nodules with smooth, straight margins, and with echogenicity similar to the thymus, suggesting intrathyroid ectopic thymus [10].

Given the need for large-scale ultrasound screenings of the thyroid gland, we recently performed ultrasound thyroid gland screening in children from three Japanese prefectures (Aomori, Yamanashi and Nagasaki Prefectures), in order to analyze the frequencies of specific ultrasound findings of the thyroid gland, with the same procedures for the ultrasound screenings as used in the Fukushima Health Management Survey, and identified thyroid cysts in 56.9% of the participants [12]. This previous report showed only the categorized results of thyroid findings: “A” (“A1” and “A2”), “B” or “C”, and was based on the crude data only [12]. It is anticipated that the detailed information presented in this report will provide greater disclosure. The current report aims to present further analyses of the results of ultrasound thyroid gland screening in children from these three Japanese prefectures.

## Materials and Methods

### Ethics Statement

This study was approved by the ethics committees of Hirosaki University, Yamanashi University and Nagasaki University, respectively. It was conducted in accordance with the guidelines expressed in the Declaration of Helsinki. Written informed consent was obtained from the parents of all surveyed children.

### Study Area

The survey was conducted in Aomori Prefecture by Hirosaki University, in Yamanashi Prefecture by Yamanashi University, and in Nagasaki Prefecture by Nagasaki University, respectively (**Figure 1**). These areas were suitable for the current investigation, since they have thyroid ultrasound specialists and medical facilities enabling further examination, and they are located far from each other. More precisely, these areas are geographically dispersed throughout the eastern, central, and western regions of Japan, and are thought to have been unaffected by radioactive material from the FNPP accident. We did not consider the level of iodine intake in each prefecture, because Japan is generally an iodine-rich area [13].

**Figure 1:** Location of Aomori Prefecture, Yamanashi Prefecture, Nagasaki Prefecture and Fukushima Prefecture.

### Study Population

Ultrasound examinations were performed between November 2012 and January 2013. To perform ultrasound examinations in many children at once, and to match the ages of the participants in the Fukushima Health Management Survey, we selected a kindergarten, an elementary school, a junior high school and a high school from each prefecture for this study. We selected these kindergartens and schools because they are located near the center of each prefecture, and furthermore agreed to participate in this study. All children aged 3 to 18 years, from each kindergarten and school, were invited to participate in the study. Because we wished to clarify the general status of the thyroid gland in children, we did not define exclusion criteria in these participants. Children whose parents refused to participate were excluded from the study. Because we emphasized that potential subjects were free to decline to participate on any grounds, we did not collect the reasons why they refused. The overall participation rate was 85.0%. In total, 4,365 children (Aomori: 1,630 children; Yamanashi: 1,366 children; Nagasaki: 1,369 children) underwent the ultrasound examinations. The characteristics of participants in the three examination areas are shown in **Table 1**. The number of children aged 3 to 4 years who were included in the study was 41 in Nagasaki, 5 in Yamanashi and 25 in Aomori, respectively. The largest group of children in all examination areas was 10 to 14 years. In total, 47.5% (2,075/4,365) of the children were male and 52.5% (2,290/4,365) were female.

**Table 1:** Characteristics of participants in the three examination areas.

	Aomori		Yamanashi		Nagasaki		All areas		Total
	(n = 1,630)		(n = 1,366)		(n = 1,369)				
Age, y	Male	Female	Male	Female	Male	Female	Male	Female	
3–4	11	14	1	4	21	20	33	38	71
5–9	181	173	148	170	210	210	539	553	1,092
10–14	352	321	295	305	295	295	942	921	1,863
15–18	239	339	154	289	168	150	561	778	1,339
Total	783	847	598	768	694	675	2,075	2,290	4,365

### Ultrasonography

In all cases, ultrasonographic examination was conducted using 7.75-MHz probes (12L-RS linear array transducer [GE Healthcare, Japan] and LOGIQ e Expert ultrasound [GE Healthcare, Japan]), which is the same equipment as that used in the Fukushima Health Management Survey [3]. The examiner in each prefecture was defined as being an expert in thyroid ultrasonography, and was someone who had experience conducting thyroid screening in the Fukushima Health Management Survey. The examination protocol was the same as in the Fukushima Health Management Survey of the Fukushima Prefecture, i.e. two or more images from each lobe (cross section and longitudinal section) were saved from all children, and the thyroid volume, structure, echogenicity, nodules, cysts, and the presence of pathologies, such as congenital abnormalities (e.g. congenital defect, ectopic thymus or ultimobranchial body) were recorded. In cases with nodules, the assessor recorded the number of nodules and the location of the largest nodule, and measured the greatest dimension of the nodules. In cases with cysts, the assessor also recorded the multifocality of the cysts and the location of the largest cyst, and measured the greatest dimension of the cysts. In cases of questionable findings, expert panels of thyroidologists from the three examination areas, together with thyroid specialists from related Japanese academic societies, discussed them and reached final agreement.

### Statistical methods

In this study, the age distribution of the study population differed from that of the standard population of Japanese children. To estimate the general frequency, the age-adjusted prevalence was calculated by using the 2010 Japan standard population distribution for children aged between 3 and 18 years [14]. We used logistic regression analysis to assess the associations between the prevalence of thyroid cysts and nodules and age, gender and the examination areas. We conducted all analyses with SAS for UNIX (SAS institute, Cary, NC). We considered *P*<0.05 to be statistically significant.

## Results

**Table 2** shows the number of cases with thyroid cysts and nodules identified by ultrasound examinations in the 3 examination areas. Overall, thyroid cysts were identified in 56.88% and thyroid nodules in 1.65% of the participants. Most cysts were small in size, with a maximum diameter of 5 mm or less. Thyroid cysts and nodules with a maximum diameter of more than 5 mm were identified in 4.58% and 1.01% of the total participants, respectively.

**Table 2:** Number of cases with thyroid cysts and nodules in the three examination areas.

			Aomori		Yamanashi		Nagasaki		All areas
		Age,y	Male	Female	Male	Female	Male	Female	Total
Cyst	All	3–4	1/11	6/14	1/1	4/4	1/21	1/20	14/71
		5–9	103/181	99/173	94/148	111/170	71/210	67/210	545/1,092
		10–14	183/352	206/321	212/295	236/305	130/295	160/295	1,127/1,863
		15–18	145/239	203/339	96/154	201/289	71/168	81/150	797/1,339
		Total	432/783	514/847	403/598	552/768	273/694	309/675	2,483/4,365 (56.88%)
	≤5 mm	3–4	1/11	6/14	1/1	4/4	1/21	1/20	14/71
		5–9	101/181	94/173	94/148	109/170	69/210	65/210	532/1,092
		10–14	171/352	188/321	199/295	218/305	121/295	145/295	1,042/1,863
		15–18	132/239	170/339	86/154	174/289	63/168	70/150	695/1,339
		Total	405/783	458/847	380/598	505/768	254/694	281/675	2,283/4,365 (52.30%)
	>5 mm	3–4	0/11	0/14	0/1	0/4	0/21	0/20	0/71
		5–9	2/181	5/173	0/148	2/170	2/210	2/210	13/1,092
		10–14	12/352	18/321	13/295	18/305	9/295	15/295	85/1,863
		15–18	13/239	33/339	10/154	27/289	8/168	11/150	102/1,339
		Total	27/783	56/847	23/598	47/768	19/694	28/675	200/4,365 (4.58%)
Nodule	All	3–4	0/11	0/14	0/1	0/4	1/21	0/20	1/71
		5–9	2/181	2/173	2/148	1/170	0/210	0/210	7/1,092
		10–14	1/352	11/321	8/295	4/305	0/295	4/295	28/1,863
		15–18	6/239	13/339	3/154	9/289	2/168	3/150	36/1,339
		Total	9/783	26/847	13/598	14/768	3/694	7/675	72/4,365 (1.65%)
	≤5 mm	3–4	0/11	0/14	0/1	0/4	0/21	0/20	0/71
		5–9	1/181	1/173	2/148	0/170	0/210	0/210	4/1,092
		10–14	0/352	4/321	5/295	2/305	0/295	1/295	12/1,863
		15–18	3/239	5/339	1/154	2/289	1/168	0/150	12/1,339
		Total	4/783	10/847	8/598	4/768	1/694	1/675	28/4,365 (0.64%)
	>5 mm	3–4	0/11	0/14	0/1	0/4	1/21	0/20	1/71
		5–9	1/181	1/173	0/148	1/170	0/210	0/210	3/1,092
		10–14	1/352	7/321	3/295	2/305	0/295	3/295	16/1,863
		15–18	3/239	8/339	2/154	7/289	1/168	3/150	24/1,339
		Total	5/783	16/847	5/598	10/768	2/694	6/675	44/4,365 (1.01%)

Data are expressed as a case number/a number of participants. A parenthesis indicates percentage in total participants. Forty-three participants had both cyst and nodule.

The maximum diameter of thyroid cysts ranged from 0.8 mm to 12.1 mm and most of the children who had cysts had 2 or more cysts (2,240/2,482, 90.25%). The prevalence of cysts varied among the examination areas (58.04% in Aomori, 69.91% in Yamanashi and 42.51% in Nagasaki), the difference being significant when adjusted for age and gender (*P*<0.001). However, no significant difference among the examination areas was observed in the prevalence of cysts with a maximum diameter of more than 5 mm adjusted for age and gender (5.09% in Aomori, 5.12% in Yamanashi and 3.43% in Nagasaki, *P*>0.2).

The maximum diameter of nodules ranged from 1.9 mm to 23.5 mm. Two or more nodules were identified in 26.39% (19/72) of nodule cases. Forty-three participants had both nodules and cysts. The prevalence of nodules varied among the examination areas (2.15% in Aomori, 1.98% in Yamanashi and 0.73% in Nagasaki), the difference being significant when adjusted for age and gender (*P* = 0.03 for Yamanashi vs. Nagasaki, *P* = 0.01 for Aomori vs. Nagasaki). However, no significant differences among the examination areas were observed in the prevalence of nodules with a maximum diameter of more than 5 mm adjusted for age and gender (1.29% in Aomori, 1.10% in Yamanashi and 0.58% in Nagasaki, *P*>0.1).

**Table 3** shows the effect of age on the prevalence of thyroid cysts and nodules. The prevalence of thyroid cysts and nodules, especially those with a maximum diameter of more than 5 mm, significantly increased with age. Females had a significantly higher prevalence of thyroid cysts and nodules with a maximum diameter of more than 5 mm than males (**Table 4**). We also estimated the prevalence of thyroid cysts and nodules adjusted for the Japanese population aged between 3 and 18 years (**Table 5**). As reflections of the small fraction of children aged 3 to 4 years and the female preponderance of the study population, the age-adjusted prevalence of thyroid cysts and nodules (52.35% for thyroid cysts and 1.54% for thyroid nodules) were found to be less than the unadjusted prevalence (56.88% for thyroid cysts and 1.65% for thyroid nodules).

**Table 3:** Number of cases with thyroid cysts and nodules according to age and the effect of age on their prevalence.

	Age, y	3–4	5–9	10–14	15–18	OR (95% CI)	*P*
		(n = 71)	(n = 1,092)	(n = 1,863)	(n = 1,339)		
Cyst	All	14	545	1,127	797	1.05 (1.03, 1.06)	<0.001
		(19.72)	(49.91)	(60.49)	(59.52)		
	≤5 mm	14	532	1,042	695	1.01 (1.00, 1.03)	0.10
		(19.72)	(48.72)	(55.93)	(51.90)		
	>5 mm	0	13	85	102	1.21 (1.16, 1.28)	<0.001
			(1.19)	(4.56)	(7.62)		
Nodule	All	1	7	28	36	1.15 (1.07, 1.25)	<0.001
		(1.41)	(0.64)	(1.50)	(2.69)		
	≤5 mm	0	4	12	12	1.08 (0.96, 1.21)	0.19
			(0.37)	(0.64)	(0.90)		
	>5 mm	1	3	16	24	1.21 (1.09, 1.34)	<0.001
		(1.41)	(0.27)	(0.86)	(1.79)		

A parenthesis indicates percentage in participants of the age category.

OR indicates odds ratio per 1 year adjusted by gender and the examination areas.

CI indicates confidence interval.

**Table 4:** Number of cases of thyroid cysts and nodules according to gender and the effect of gender on their prevalence.

		Male	Female	OR (95% CI)	*P*
		(n = 2,075)	(n = 2,290)		
Cyst	All	1,108 (53.40)	1,375 (60.04)	1.25 (1.10, 1.41)	<0.001
	≤5 mm	1,039 (50.07)	1,244 (54.32)	1.14 (1.01, 1.28)	0.04
	>5 mm	69 (3.33)	131 (5.72)	1.61 (1.19, 2.17)	0.002
Nodule	All	25 (1.20)	47 (2.05)	1.55 (0.95, 2.55)	0.08
	≤5 mm	13 (0.63)	15 (0.66)	0.96 (0.45, 2.02)	0.90
	>5 mm	12 (0.58)	32 (1.40)	2.19 (1.12, 4.29)	0.02

A parenthesis indicates percentage in participants of the gender category.

OR indicates odds ratio of female compared to male as a reference adjusted by age and the examination areas.

CI indicates confidence interval.

**Table 5:** Age-adjusted prevalence of thyroid cysts and nodules.

		Male % (95%CI)	Female % (95%CI)	Total % (95%CI)
Cyst	All size	48.52 (46.27, 50.78)	55.76 (53.28, 58.23)	52.35 (50.64, 54.06)
	≤5 mm	45.69 (43.43, 47.95)	51.10 (48.60, 53.59)	48.52 (46.27, 50.78)
	>5 mm	2.83 (2.17, 3.50)	4.66 (3.88, 5.44)	3.82 (3.30, 4.34)
Nodule	All size	1.39 (0.60, 2.19)	1.67 (1.19, 2.14)	1.54 (1.09, 1.99)
	≤5 mm	0.57 (0.26, 0.89)	0.53 (0.26, 0.81)	0.55 (0.35, 0.76)
	>5 mm	0.82 (0.09, 1.55)	1.13 (0.74, 1.53)	0.99 (0.59, 1.39)

The estimated prevalence is age-adjusted to the 2010 Japan standard population.

CI indicates confidence interval.

Ultrasound findings other than cysts and nodules are shown in **Table 6**. The most frequent finding was ectopic thymus. The percentage of ectopic thymus decreased with age. Diffuse goiter, ultimobranchial body, lymph node swelling and thyroid agenesis were identified in participants aged 5 years or older.

**Table 6:** Number of cases with ultrasound findings other than cysts and nodules.

Age, y	3–4	5–9	10–14	15–18	Total
	(n = 71)	(n = 1,092)	(n = 1,863)	(n = 1,339)	(n = 4,365)
Ectopic thymus	4 (5.63)	49 (4.49)	30 (1.61)	2 (0.15)	85 (1.95)
Diffuse goiter	0	10 (0.92)	32 (1.72)	19 (1.42)	61 (1.40)
Ultimobranchial body	0	10 (0.92)	12 (0.64)	10 (0.75)	32 (0.73)
Lymph node swelling	0	1 (0.09)	6 (0.32)	2 (0.15)	9 (0.21)
Thyroid agenesis	0	1 (0.09)	1 (0.05)	0	2 (0.05)

A parenthesis indicates percentage in participants of the age category.

## Discussion

Few reports have studied the prevalence, spectrum of appearance and management of ultrasound-detected findings in the thyroid glands of children, except for screening programs conducted around Chernobyl [5]. Within the framework of the Chernobyl Sasakawa Medical Cooperation Project, ultrasound examination of the thyroid gland was conducted around Chernobyl in Ukraine, the Russian Federation and Belarus between 1991 and 1996 [5]. In this project, 120,605 children were examined at five centers in three countries, and 63 cases with thyroid cancer (0.052%) were identified. Of note, 38 cases (0.192%) of thyroid cancer were identified in the Gomel region (Belarus), which was the area that was most contaminated by the accident. Also, this study revealed that 42,470 (35.9%) children showed increased thyroid volume (goiter), ranging from 18% to 54% in the five examination centers [5]. This relatively high frequency of goiter reflected the iodine deficient status of this area during the study period [11], [13]. On the other hand, only 502 (0.42%) showed cystic lesions, ranging from 0.19 to 0.63% at the five examination centers, which were much lower frequencies than those observed in our current study. Further, in 2000, we conducted ultrasound examinations of the thyroid gland in 250 Japanese schoolchildren in Nagasaki (Japan) and observed the presence of goiters in only 4 cases (1.60%), while 2 cases (0.80%) had cystic degeneration and a single thyroid cyst, and no cases had thyroid nodules [13]. Of course, a big difference of detection sensitivity and image quality of ultrasound machine at the different time and place of examination should be deeply considered and a standardized method and protocol of ultrasound examination such as common diagnostic criteria should be implemented.

In the current study, we conducted ultrasound examination of the thyroid gland in 4,365 Japanese children (from Aomori, Yamanashi and Nagasaki) in 2013 and identified thyroid cysts in 56.88% and thyroid nodules in 1.65% of them, learning from the same method and protocol of the Fukushima Health Management Survey. Following the first report that aimed at a rapid announcement of the crude data according to sociomedical needs [12], our current further study added the new information. For instance, the prevalence of cysts with a maximum diameter of smaller than 5 mm varied among the examination areas, and the most frequent finding other than cysts was ectopic thymus which showed a decreased prevalence with age.

Focusing only on the subset data of Nagasaki in the current study, we identified thyroid cysts in 42.51% and thyroid nodules in 0.73% of the children, which indicates a gap in the frequencies of thyroid cysts and nodules between the studies conducted in 2000 [13] and 2013 (the current study). These gaps between studies could be mainly due to the dramatic advances in ultrasound technology, including imaging quality. New ultrasound technologies, such as digital beam formers, tissue harmonic imaging and speckle reduction have greatly improved the image quality of diagnostic ultrasound machines [15]. These advances enable us to perform detailed evaluation of the thyroid gland by ultrasonography, and consequently could have resulted in the relatively high observed frequency of thyroid cysts in our study, since most of the cysts we detected were less than 5 mm in diameter. In other words, if ultrasound technology advances further, there is a possibility that much more small cysts could be pointed out in the future screening.

The prevalence of both thyroid cysts and nodules varied among the three examination areas, although no significant differences were observed in the prevalence of thyroid cysts and nodules with a maximum diameter of more than 5 mm. This suggests that the differences in the frequency of thyroid cysts and nodules among the three examination areas were due to different frequencies in relatively small thyroid cysts and nodules, which were perhaps affected by inter-observer differences.

The thyroid ultrasound examination performed in the Fukushima Health Management Survey [3] targeted all prefectural inhabitants who were between 0 and 18 years of age on 11 March 2011 (approximately 360,000 inhabitants). The information released by Fukushima Prefecture indicated that 74,216 (42.56%) of the 174,376 children who underwent thyroid ultrasound examination showed thyroid cysts and 2,014 (1.15%) showed thyroid nodules [16]. Our sample size was much more limited, but the frequency of thyroid cysts and nodules was relatively high in our study, when compared with the data presented in the Fukushima Health Management Survey (56.83% vs. 42.56% for cysts and 1.65% vs. 1.15% for nodules). Since we used the same ultrasonography as was used in the Fukushima Health Management Survey, other factors, such as age composition, inter-observer differences, iodine intake of each region, socio-ecological status and family history or past history of each study participants may associate with the differences between studies. Further analysis, such as comparison with other conducting around Chernobyl or other region with the latest ultrasound machines will be needed.

In this study, we observed 85 (1.95%) cases with ectopic thymus. Furthermore, the percentage of ectopic thymus decreased with age. The thymus originates from the 3^rd^ pair of branchial pouches, with a rudimentary portion arising from the 4^th^ pair, and descends to the superior mediastinum. Anomalies of migration can cause an ectopic thymus along the path of descent. The descents of the thymus and thyroid are closely related because of the proximity of the thyroid diverticulum and the 3^rd^ branchial pouch [10], [17]. Thymic tissue can therefore get sequestered within the thyroid, giving rise to an intrathyroid ectopic thymus. The criterion for ectopic thymus in this study was “Intrathyroid lesions showing hypoechogenicity with multiple linear echogenic branching structures or punctate echogenic foci” [18], which is identical with the criterion of the Fukushima Health Management Survey [3]. On the other hand, discrimination of ultrasonographic findings between ectopic thymus and thyroid nodule, especially for papillary thyroid cancer, is sometimes difficult, and the lack of knowledge has even led to unnecessary thyroid resection [16], [19]. When evaluating ultrasound findings of the thyroid gland, especially malignancies in children, careful observation is necessary to rule out the possibility of ectopic thymus.

A large-scaled sample number was the strength of the current study even though the number was relatively small compared with the Fukushima Health Management Survey [3]. There are several limitations to this study. The current study could not include 0 to 2 year old children. Further, the number of study participants aged 3 to 4 years was much smaller than other age groups. We also could not evaluate autoimmunity of the thyroid gland or iodine intake, both of which strongly influence the ultrasound findings of the thyroid gland. Although Japan is generally an iodine-rich area due to the Japanese diet which contains a large amount of seafood, changes in diet in children may affect iodine uptake in the three examination areas. A further follow-up study is definitely needed in order to evaluate the prognosis of the thyroid cysts and nodules obeserved in childhood.

In conclusion, we conducted a sophisticated ultrasound examination of the thyroid glands of children from three Japanese prefectures besides Fukushima, and identified thyroid cysts in 56.88% and thyroid nodules in 1.65% of them, respectively. All the inhabitants of Fukushima Prefecture aged 0 to 18 years on March 11, 2011 (approximately 360,000 inhabitants) will undergo thyroid ultrasound examination every 2 years until the age of 20 years, and every 5 years thereafter [3]. The reference data observed in the current study and the further data analyses (including follow-up surveys) of children in general, can provide relevant information for the Fukushima Health Management Survey when followed up in the future through additional population studies.
